# Prevalence of Workplace Violence Against Healthcare Workers During the COVID-19 Pandemic: A Systematic Review and Meta-Analysis

**DOI:** 10.3389/fpsyg.2022.896156

**Published:** 2022-05-30

**Authors:** Zhian Salah Ramzi, Proosha Warzer Fatah, Asghar Dalvandi

**Affiliations:** ^1^College of Nursing, Sulaimani University, Sulaymaniyah, Iraq; ^2^Directory of Health of Sulaimani, Sulaymaniyah, Iraq; ^3^School of Nursing and Midwifery, Tehran Medical Sciences Branch, Islamic Azad University, Tehran, Iran

**Keywords:** healthcare worker, violence, workplace violence, systematic review, COVID-19

## Abstract

**Background:**

A large number of anxious and concerned people refer to health centers during the COVID-19 pandemic, increasing the workload of healthcare workers (HCWs) and violence against these professionals. The present study aimed to estimate the prevalence of workplace violence (WPV) against HCWs during the COVID-19 pandemic.

**Methods:**

This systematic review and meta-analysis was conducted via searching in databases such as Scopus, PubMed, and Web of Science, and observational articles reporting the prevalence of WPV against HCWs were selected. Heterogeneity between the studies was assessed using Cochran's Q test. A random-effects model was used to estimate the prevalence of WPV. Data analysis was performed in the Stata software version 16.

**Results:**

In the initial search, 680 articles were identified and screened based on the Preferred Reporting Items for Systematic Review and Meta-Analysis (PRISMA) steps. In total, 17 studies with a sample size of 17,207 HCWs were analyzed. The total prevalence of violence was estimated at 47% (95% CI: 34–61%). In addition, the prevalence of physical and psychological violence was 17% (95% CI: 6–28%) and 44% (95% CI: 31–57%), respectively. The prevalence of WPV was higher among physicians (68%; 95% CI: 31–95%) compared to other HCWs. The WPV in the America and Asia was 58 and 44%, respectively.

**Conclusion:**

According to the results, WPV against nurses is prevalent during the COVID-19 pandemic, and intervention measures are required to protect the nursing staff against such violence.

## Introduction

The COVID-19 pandemic imposed unprecedented pressure on the entire healthcare system and caused multiple challenges for healthcare workers (HCWs) (Alameddine et al., 2021). Due to long working hours, insufficient access to personal protective equipment, fear of virus transmission, and stress about moral and ethical decisions in prioritizing care, HCWs have suffered tremendous stress and anxiety, which affect their mental health (Braquehais et al., 2020; Ruiz-Fernández et al., 2020). In addition to the fear of infection, the COVID-19 pandemic has created a worst-case scenario for the HCWs who have been repeatedly attacked, humiliated, and verbally abused due to the fear of disease transmission (Belbase et al., 2021).

Workplace violence (WPV) refers to the use of force against an individual or group of people in the workplace, which leads to physical and psychological injury and even death (Ferri et al., 2016). WPV against HCWs is so common that it is recognized as a global warning phenomenon (Yenealem et al., 2019). WPV is associated with decreased job satisfaction and productivity, low quality of life, increased stress, burnout, and sleep disorders (Isaksson et al., 2008; Wu et al., 2014; Copeland and Henry, 2018; Yang et al., 2018; Zhao et al., 2018), and has a negative impact on the quality of care provision (Eneroth et al., 2017). In the first 6 months of the COVID-19 pandemic, more than 600 cases of intimidation and stigma against nurses were reported in 40 countries. The incident was most likely only the “tip of the iceberg”, and many of these incidents have not been reported for various reasons (Ghareeb et al., 2021). Therefore, some humanitarian organizations have urged governments to protect HCWs during the COVID-19 pandemic by enacting laws, creating safer work conditions, providing mental health assistance, and combating misinformation (Devi, 2020).

Studies have reported the prevalence of WPV against health professionals to be 8.4–88.3% (Lafta et al., 2021; Özkan Sat et al., 2021). Due to different results in this regard, this systematic review and meta-analysis aimed to estimate the overall prevalence of WPV against HCWs.

## Materials and Methods

This systematic review and meta-analysis was performed based on the Preferred Reporting Items for Systematic Review and Meta-Analysis (PRISMA) guideline.

### Search Strategy

To find studies regarding the prevalence of WPV against health professionals, we searched databases such as Scopus, PubMed, and Web of Science during January 2020–January 2022. The search terms were “workplace violence” OR “violence” OR “aggression” OR “bullying” OR “workplace violenc^*^” OR “violenc^*^” OR “assaul^*^” OR “assaultive behavior” OR “aggression^*^” OR “abuse” OR “bullying” OR “harassment” AND “COVID-19” OR “SARS-CoV-2” OR “COVID 19” OR “2019-nCoV” OR “coronavirus disease-19” OR “SARS CoV 2” OR “2019 novel coronavirus” OR “Wuhan coronavirus” OR “SARS Coronavirus 2” OR “Wuhan seafood market pneumonia virus” AND “health personnel” OR “physicians” OR “nurses” OR “health personnel” OR “health care provider^*^” OR “healthcare worker^*^” OR “health care professional^*^” OR “nurse^*^” OR “nursing personnel^*^” OR “registered nurse^*^” OR “physician^*^”. The reference lists of the retrieved articles were also reviewed for access to more articles.

### Inclusion and Exclusion Criteria

The inclusion criteria of the study were observational studies, studies conducted during the COVID-19 pandemic, and reporting the prevalence rate/frequency of WPV against HCWs or providing sufficient data for the calculation of this rate.

### Data Extraction

After reviewing the retrieved studies, data were extracted on the authors' name, year of publication, country, sample size, mean age of participants, and prevalence of WPV (general, physical, and non-physical violence) were extracted and recorded in a prepared form.

### Quality Appraisal

At this stage, the two authors independently examined the methodological quality of the selected studies based on the items of the STROBE checklist. In reviewing the quality of the articles, the focus was on 10 items, including the title and abstract, objectives and hypotheses, research context, inclusion criteria, sample size, statistical methods, descriptive data, interpretation of findings, research limitations, and financing. Based on each item, the articles were given a score of zero or one. The overall score was within the range of 0–10, with scores ≥6 confirming high methodological quality (Dehvan et al., 2021).

### Statistical Analysis

The prevalence rate of WPV against HCWs was calculated using a random-effects model. To visualize the heterogeneity between the studies, a forest plot was used, which reported the prevalence rate at 95% confidence interval for each study, as well as the pooled prevalence of the combined studies. In addition, statistical heterogeneity across the studies was investigated using Cochran's Q test at the significance level of <0.1 and the *I*^2^ index, based on which the values of 25, 50, and 75% indicated low, medium, and high heterogeneity, respectively (Higgins and Thompson, 2002). Subgroup analysis was also performed based on the type of the HCWs (physician, nurse, combination of professional groups) and continent (Asia and others) to investigate the potential sources of heterogeneity between the subgroups. The correlation between the prevalence of WPV with age and sample size was assessed using meta-regression analysis. Possible publication bias was also evaluated using Egger's linear regression test. Data analysis was performed in the Stata software version 16 at the significance level of *P* < 0.05.

## Results

### Study Selection

Figure 1 depicts the process of selecting, identifying, and including studies based on the PRISMA flow diagram. The initial search in Scopus, PubMed, and Web of Science resulted in 680 articles, 375 of which were duplicates and eliminated. The two authors reviewed the titles and abstracts of these articles independently. At this stage, 286 irrelevant articles (qualitative studies, letters to the editor, and review studies) were also eliminated, and 19 articles remained for further analysis. After reviewing the full text of the remaining articles, two cases were eliminated since they did not report the prevalence of violence. Finally, 17 articles were selected for the final review (Figure 1).

**Figure 1:** Flowchart of article selection.

The selected studies (*n* = 17) were performed on 17,207 medical staff. Their sample size was within the range of 67–10,516, and the largest sample size was in the study by Xie et al. (2021). Three studies had a sample size of over 1,000 (Bitencourt et al., 2021b; Xie et al., 2021; Yang et al., 2021). Nine studies were conducted in Asia (China, Iraq, Iran, Lebanon, Jordan, and Turkey), five studies were conducted in the Americas (USA, Mexico, Brazil, and Peru), one study was conducted in Egypt, and one study was performed in Belgium. The selected studies had high methodological quality. Table 1 shows the most important findings of the reviewed studies.

**Table 1:** Characteristics of reviewed studies.

**References**	**Sample size**	**Country**	**Workplace violence (WPV) Prevalence (%)**			**Results**
			**Physical**	**Verbal**	**Total**	
Alameddine et al. (2021)	265	Lebanon	-	-	74.7	**Target group:** Nurses
						The majority of the nurses were female (64.9%), aged 30–45 years (75.8%), and married (68.7%). Mean resilience score of the nurses who had never experienced WPV was higher than those reporting WPV.
Arafa et al. (2021)	104	Egypt	9.6	42.6	-	**Target group:** Nurses
						The study was performed on nurses and physicians, and nurses' data were extracted separately.
Byon et al. (2021)	373	USA	44.4	67.8	-	**Target group:** Nurses
						Most of the nurses were female (94.4%), aged <40 years (62.7%), and had at least 3 years of nursing experience (85.5%). The nurses who provided care to COVID-19 patients experienced more physical violence (aOR: 2.18; 95% CI: 1.30–3.67) and verbal abuse (aOR: 2.10; 95% CI: 1.22–3.61) than those who did not provide care to these patients.
Khatatbeh et al. (2021)	225	Jordan	-	31.1	19.6	**Target group:** Nurses
						Mean age of the nurses was 32.5 years, and the majority were female (94.2%) and married (82.7). Exposure to violence was one of the predictors of quality of life and burnout in the nurses.
Özkan Sat et al. (2021)	263	Turkey	8.4	57.8	-	**Target group:** Nurses
						Mean age of the nurses was 31.2 ± 7.1 years, 88.2% were female, and 63.9% had a bachelor's degree.
Bitencourt et al. (2021a)	180	Brazil	-	-	51.1	**Target group:** Nurses
						Single nurses, nursing assistants, those with a history of COVID-19, those who had been in contact with COVID-19 patients, and those who experienced violence before the COVID-19 pandemic were more likely to experience violence than other HCWs.
Ghanbari et al. (2020)	112	Iran	17.8	62.5	-	**Target group:** Nurses
						Most of the nurses were female (94%) and married (78%). Mean age and mean work experience of the nurses were 33.11 ± 5.22 and 4.55 ± 5.26 years, respectively. Psychological violence was mostly inflicted by patient companions, and physical violence was mostly inflicted by patients.
Aspera-Campos et al. (2020)	562	Mexico	12.8	-	47.7	**Target group:** Nurses
						Nurses were more exposed to violence than other HCWs (*P =* 0.018). Female gender and being a nurse increased the risk of exposure to WPV 2.5 and 3 times, respectively (rate of mixed violence: 34.9%).
Buran and Altin (2021)	67	Turkey	-	23.9	-	**Target group:** Physicians
						Mean age of the participants was 34.7 ± 9.2 years. Most of the physicians were female (61.2%), married (61.2%), and had children (55.2%). Rate of violence was higher in the emergency department physicians compared to the other departments (*P =* 0.018).
Ghareeb et al. (2021)	382	Jordan	-	52	65.5	**Target group:** Physicians and nurses. Most of the participants were female (57.6%) and aged 35–50 years (47.1%). Prevalence of verbal and mixed violence was 52 and 32%, respectively. The most common verbal violence was shouting (90.5%) and threat of harm (58.6%).
Lafta et al. (2021)	505	Iraq	-	-	88.3	**Target group:** Physicians
						Most of the physicians were aged <30 years (44%) and female (61.4%). Violence was mostly perpetrated by patients' families and relatives (72.4%).
Muñoz Del Carpio-Toia et al. (2021)	200	Peru	-	-	84.5	**Target group:** Physicians Mean age of the participants was 37.5 years (rang: 25–47 years). Rate of mixed violence was 84.5%. Female gender (OR: 2.48; 95% CI: 1.06–5.83) and working in the COVID-19 ICU (OR: 5.84; 95% CI: 1.60–21.28) were the most significant risk factors for WPV.
Somville et al. (2021)	196	Belgium	-	-	32	**Target group:** Physicians
						More than half of the physicians were aged more than 40 years, and 42% were emergency physicians.
Wang et al., 2020	1,063	China	-	-	20.4	**Target group:** HCWs HCWs who experienced violence were more likely to have mental disorders than those who did not.
Xie et al. (2021)	10,516	China	8.4	15.8	18.5	**Target group:** Mental health professionals
						A correlation was observed between male gender (OR: 1.42; *P* < 0.01), care provision to COVID-19 patients (OR: 3.10; *P* < 0.01), severe anxiety symptoms (OR: 1.12; *P* < 0.01), and WPV.
Bitencourt et al. (2021b)	1,166	USA	-	-	49.4	**Target group:** Physician, nurses, and assistant nurses.
						Most of the participants were female (75.3%) and aged <40 years (61.66%).
Yang et al. (2021)	1,028	China	-	-	20.4	**Target group:** HCWs
						The majority of the respondents were female (66.6%), highly educated (93.7%; bachelor's degree or above), and married (72.1%). WPV was an independent predictor of stress.

The obtained results indicated that the pooled prevalence of physical and non-physical violence was 17% (95% CI: 6–28%) and 44% (95% CI: 31–57%), respectively. In total, 13 studies reported the prevalence of total violence with the pooled prevalence of 47% (95% CI: 34–61%) (Figure 2). In these studies, violence was reported against nurses, physicians, or both of these groups together.

**Figure 2:** Forest plots of prevalence of WPV among HCWs during COVID-19 pandemic.

The results of the subgroup analysis showed that the prevalence of general WPV was 47% among nurses (95% CI: 30–65%), 68% among physicians (95% CI: 31–95%) and 35% among both of these groups together (95% CI: 16–53%). Also, the pooled prevalence of WPV against HCWs in studies conducted in Asia and the America was 44% (95% CI: 23–64%) and 58% (95% CI: 42–74%), respectively.

On the other hand, the results of meta-regression analysis showed no correlation between the prevalence of violence with the sample size and mean age of HCWs. Egger's tests were separately performed regarding the meta-analysis (total violence; *P* = 0.812), physical violence (*P* = 0.420), and non-physical violence (*P* = 0.413), none of which were considered significant (Figure 3).

**Figure 3:** Publication bias for total violence.

## Discussion

To the best of our knowledge, this is the first study to estimate the pooled prevalence of WPV against HCWs during the COVID-19 pandemic. With the rapid spread of the COVID-19 pandemic, people have become physically isolated, restricted in their social interactions, and feel intimidated by those who are infected or are in close contact with COVID-19 patients (Abuhammad et al., 2020). HCWs are constantly at the risk of the disease due to direct contact with COVID-19 patients, which has increased people's sensitivity and provoked violent reactions toward these professionals. A study indicated that nurses in Mexico are assaulted while going to work, while a Filipino nurse was attacked with bleach and suffered eye damage. Specialists are also chased by thugs and even neighbors and landlords and threatened to evacuate their homes (CDT., 2020; Economist., 2020; McKay et al., 2020; Semple, 2020).

According to the International Committee of the Red Cross (ICRC), more than 600 cases of violence against HCWs occurred in the first 6 months of the pandemic (Devi, 2020). Health professionals were exposed to WPV even before the COVID-19 pandemic. In their meta-analysis, Liu et al. reported that 26.8 and 44.9% of HCWs experience physical and non-physical violence every year (Liu et al., 2019). In the present study, the overall prevalence of WPV against HCWs was estimated at 47%, and the prevalence of physical and non-physical violence was 17 and 44%, respectively. The sudden onset of COVID-19 surprised the healthcare system, and as the disease spreads rapidly, large numbers of patients are referred to healthcare facilities. Inadequate environments and crowded emergency departments could cause stress and frustration in healthcare providers (especially physicians and nurses), as well as patients and their families, thereby increasing the risk of violence (Medley et al., 2012). In some studies, only violence in general was examined with one question. In some studies, violence was divided into two types, physical (hitting, pinching, biting, scratching, chocking, and hair-pulling) and psychological **(**cursing, yelling, name-calling, and insulting).

Patient-related factors such as acute illness, fear of unpredictability, and severe stress could lead to violence against HCWs (Stene et al., 2015). In another study, the insufficient number of medical staff and unmet patient demands were reported to be the main causes of aggression against HCWs (Al Anazi et al., 2020). In Central America and the Caribbean, physicians and nurses have been attacked on several occasions due to frustration with the lack of proper care and reluctance to follow the burial rules of COVID-19 patients (Bhatti et al., 2021). Byon et al. (2020) conducted a meta-analysis to estimate the prevalence of WPV against HCWs and systematically reviewed articles published during 2005–2019. The findings showed that the overall prevalence of WPV was 22.3%, and the prevalence of physical and non-physical violence was 10.2 and 36.4%, respectively. The prevalence of WPV in the current pandemic seems to be increasing compared to the past. Findings by continent show that the prevalence of general WPV in America was higher than in Asia. The reason for this finding can be attributed to the cultural characteristics and context of these communities. In the COVID-19 pandemic, although similar precautions were taken in all countries, because violence is a phenomenon influenced by culture and context, the prevalence of WPV varied from region to region.

In the present study, no correlations were observed between the prevalence of WPV, the mean age of HCWs, and the sample size of the reviewed studies. Therefore, it could be concluded that WPV affects all healthcare providers regardless of age and may be considered another pandemic during the COVID-19 outbreak. One of the limitations of this meta-analysis was the possibility of recall bias in the earlier studies. Furthermore, all the reviewed studies were based on the reports of HCWs for measuring violence, which is a potential source of self-report bias and may underestimate the actual prevalence rate of WPV. The last limitation was that selected studies did not specify whether the violence against HCWs was perpetrated by patients or their caregivers. Therefore, this idea should not come to mind that violence during treatment of COVID-19 patients is an everyday phenomenon.

## Conclusion

According to the results, WPV against HCWs is highly prevalent during the COVID-19 pandemic and may lead to physical and psychological issues in healthcare professionals and even affect the quality of the provided care. Therefore, it is critical to take protective measures in hospitals and medical centers and provide training to HCWs on the proper management of aggressive patients and stress.

### Implications for Nursing Management

The high prevalence of violence against healthcare workers deprives the possibility of providing desirable nursing care and in addition to causing psychological disorders in healthcare workers and reducing their quality of life, it can also endanger patients' lives by increasing the risk of medication errors. In this epidemic, healthcare workers were exposed to violence inside and outside the hospital. It is necessary to take measures to protect them so that in similar crises, healthcare workers who are always at the forefront can be supported and protected.

## Data Availability Statement

The original contributions presented in the study are included in the article/supplementary material, further inquiries can be directed to the corresponding author.

## Author Contributions

ZSR and PWF conceived the idea, participated in data extraction, analysis, and draft writing. AD and ZSR participated in analysis, manuscript preparation, and revision. All authors read and approved the final version of the manuscript to be considered for publication.

## Conflict of Interest

The authors declare that the research was conducted in the absence of any commercial or financial relationships that could be construed as a potential conflict of interest.

## Publisher's Note

All claims expressed in this article are solely those of the authors and do not necessarily represent those of their affiliated organizations, or those of the publisher, the editors and the reviewers. Any product that may be evaluated in this article, or claim that may be made by its manufacturer, is not guaranteed or endorsed by the publisher.

## Abbreviations

HCW: healthcare workers
PRISMA: Preferred Reporting Items for Systematic Review and Meta-Analysis
WPV: workplace violence.
